The article "MiR-16-5p inhibits breast cancer by reducing AKT3 to restrain NF-κB pathway" was retracted in 2022. Reasons: duplicated images; signs of a paper mill.

# MiR-16-5p inhibits breast cancer by reducing AKT3 to restrain NF-κB pathway

**DOI:** 10.1042/BSR20191611

**Published:** 2019-08-23

**Authors:** Liwei Ruan, Xiaojun Qian

**Affiliations:** Department of Breast and Thyroid Surgery, Shaoxing People’s Hospital, Shaoxing Hospital of Zhejiang University, Shaoxing 312000

**Keywords:** AKT3, breast cancer, metastasis, miRNA, NF-κB

## Abstract

**Background:** Breast cancer endangers the life of women and has become the major cause of deaths among them. MiRNAs are found to exert a regulatory effect on the migration, proliferation and apoptosis of breast cancer cells. This research aims at investigating the miR-16-5p expression and its effect on the pathogenesis of breast cancer. **Methods:** Their clinical data were analyzed with qRT-PCR. CCK8, EdU and Transwell was performed to explore the function of miR-16-5p in cell migration and proliferation of breast cancer cells. Dual-luciferase reporter assay, immunohistochemistry and Western blotting were carried out to explore the relation between miR-16-5p and AKT3. **Results:** It was discovered that miR-16-5p was lowly expressed in breast cancer patients. Meanwhile, breast cancer patients with under-expressed miR-16-5p had a lower survival rate than those with highly expressed miR-16-5p. Furthermore, decreased miR-16-5p in cell and animal models enhanced migration and proliferation of breast cancer cells, stimulated cell cycle and reduced cell apoptosis. Finally, we found miR-16-5p restrained the NF-κB pathway and decreased *AKT3* gene, thereby suppressing the breast cancer development. **Conclusion:** It can be seen that miR-16-5p exhibits a low expression in breast cancer tissues, which can inhibit breast cancer by restraining the NF-κB pathway and elevating reducing AKT3.

## Introduction

As the most common tumor, breast cancer is still an issue to be resolved in the world [1]. According to the global cancer statistics, there were more than 1.7 million new cases of breast cancer in 2012, taking up 25% of the incidence rate of all cancers [2]. In spite of these depressed statistics, advanced diagnosis methods, introduced molecular gene signature platforms and breast cancer management contribute to more effective treatment and regulation strategies, thus reducing the mortality rate of breast cancer [3]. However, in consideration of the difficulty in treating metastatic and/or intractable tumors as well as the high mortality rate, there is still a need for a large quantity of studies regarding this field [4–6]. In spite of progresses in systemic chemotherapy, patients with metastatic breast cancer still have a median survival of less than 2 years [7]. Therefore, besides the surgical treatment, radiotherapy, chemotherapy and immunotherapy of existing breast cancer treatments, scientific research workers need to explore more effective ways to diagnose breast cancer early, predict the prognosis of breast cancer, inhibit breast cancer metastasis, and reduce the mortality of patients with breast cancer.

The article "MiR-16-5p inhibits breast cancer by reducing AKT3 to restrain NF-κB pathway" was retracted in 2022. Reasons: duplicated images; signs of a paper mill.

MiRNA, discovered in eucaryon, is a type of non-coding RNA molecules, with the length of approximately 22–25 nt. It is able to pair with complementary bases to identify and directly degrade the target genes and inhibit their translation, thus realizing post-transcriptional regulation [8,9]. The miRNA is first described in nematodes and is highly conservative among humans, plants and viruses. The function of protein-coding genes in the tumors instead of the potential roles of miRNA in tumors has been emphasized in research in the past two decades, but miRNAs exert crucial effects in the development of such malignant tumors as osteosarcoma, esophageal cancer and lung cancer according to studies in recent years [10–12]. Moreover, miRNAs act on various target protein genes, so as to be involved in each link of the tumor metastasis regulation. Besides, they are capable of activating tumor metastasis [13,14] and suppressing it at the same time [15,16]. Therefore, the miRNA is considered as a novel specific biomarker for tumor metastasis as well as a target for treatment, thus providing a basis for diagnosing and treating breast cancer metastasis.

Recent research of some scholars at home and abroad have demonstrated that miRNAs exert a pivotal effect on the mechanism of breast cancer [17,18]. Cai et al. [19] found that SNHG16 competitively binds to miR-98 with E2F5, thus stimulating the migration of breast cancer cells. Wei et al. [20] found that miR-223 acts as a potential tumor marker and inhibits FOXO1 in breast cancer. However, at present, the study on breast cancer is still at the beginning level of random selection of a miRNA, which is still not rigorous on the basis of the establishment. Deep study of miRNA expression difference in breast cancer will lay a solid foundation for the diagnosis and treatment of breast cancer.

## Materials and methods

### Specimen collection and processing

Seventy-two pairs of breast cancer and adjacent noncancerous tissues undergoing surgery and confirmed by pathology were collected. The fresh tissues were removed from lesions and adjacent noncancerous tissues using the special forceps, immediately after which they were rinsed with DEPC and placed into the refrigerated tube by a professional physician, and the liquid nitrogen tank was labeled for freezing. Then the clinical data were collected in the Department of Pathology. The whole process was approved by the patients and authorized by the Ethics Committee of Shaoxing People’s Hospital.

The article "MiR-16-5p inhibits breast cancer by reducing AKT3 to restrain NF-κB pathway" was retracted in 2022. Reasons: duplicated images; signs of a paper mill.

### Cell culture and transfection

BT-549 and MCF-7 cells (Shanghai Cell Bank of the Chinese Academy of Sciences) were cultured with RPMI 1640 medium with 10% inactivated FBS, 100 μ/ml penicillin and 100 μ/ml streptomycin. The medium would be replaced once every 2 or 3 days. Cell passage began when the cell fusion degree reached 90% to maintain the cells in the logarithmic growth phase for subsequent experiments. The miR-16-5p mimics and NCs were bought from GenePharma (Shanghai, China). All transfection assays were carried out using Lipofectamine 2000 Reagent (Invitrogen, CA, U.S.A.) with reference to the manufacturer’s instructions.

### Cell proliferation

Cells were seeded on a 96-well plate and incubated for 1 h by CCK8 (Beyotime, Nantong, China). Then the absorbance at 450 nm was calculated using the TECAN infinite M200 Multimode microplate reader (Tecan, Mechelen, Belgium). After that, the EDU assay was conducted to examine the proliferation of cells. The same experiment was carried out for three times.

### Cell migration

MiR-16-5p mimics, inhibitors and NCs were applied to transfect the cells inoculated on a six-well plate. Approximately 100 μl cell suspension with serum-free medium was added into the upper chamber, and 600 μl medium with 10% FBS into the lower chamber. After 36 h of transfection, the cells were stained with Crystal Violet staining solution (Beyotime, Nantong, China) and counted, and six fields of view were selected in each well for photographing under ×40 magnification. The same experiment was carried out for three times.

### Detection of cell cycle

Cells in the logarithmic growth phase in transfection group were subjected to flow cytometry. They were inoculated on to a six-well plate at the density of 1 × 10^5^/well and cultured for 24 h. After digestion with trypsin, the cells were collected, washed three times with pre-cooled PBS, fixed with ethanol and cultured overnight at 4°C. Subsequently, the cells were added with iodides and stained for 25 min away from light. Finally, flow cytometry was adopted to examine the cell cycle in each transfection group, and the experiment was repeated three times for averaging.

### Determination of cell apoptosis

Cells were digested with trypsin, collected and prepared into single cell suspension, followed by washing twice with pre-cooled PBS with the cell density adjusted to 1 × 10^6^/ml. Then the cells in each tube were added with 100 μl single cell suspension and 10 μl Annexin-V for 15 min of incubation at 4°C in the dark. Following the addition of 380 μl buffer, 10 μl PI was added to each tube, immediately after which flow cytometry analysis was conducted. Ultimately, the cells were transfected with miRNA mimics and inhibitors (Gemma, Shanghai, China) using Lipofectamine 2000.

The article "MiR-16-5p inhibits breast cancer by reducing AKT3 to restrain NF-κB pathway" was retracted in 2022. Reasons: duplicated images; signs of a paper mill.

### Immunohistochemistry

Three pairs of breast cancer and adjacent noncancerous tissue sections were selected, followed by H&E staining. Then the immunohistochemical staining was performed via streptomycin affinity-peroxidase (s-p) method based on the standard procedures. The cells stained with AKT3, P50 and P65 were in the nucleus and/or cytoplasm, after which they turned brownish yellow or tan.

### Animal experiment

BALB/c nude mice received subcutaneous injections of 1 × 10^6^ MCF-7 cells and BT-549 cells (miR-16-5p inhibitor or negative control). Experimental operations in the present study gained the consent from the Ethics Committee for Experimental Animals in Shaoxing People’s Hospital. Animal experiments took place in SPF Animal Laboratory at Shaoxing University.

### qRT-PCR

Based on the TRIzol Total RNA manual, centrifugation was performed at 4°C, and isopropanol precipitates in the upper aqueous phase were harvested, rinsed and dried at room temperature. Subsequently, 20–30 ml DEPC was added, RNA concentration was calculated and RNAs were preserved in a refrigerator at −80°C. With reference to instructions of the Takara OneStep PrimeScript® miRNA cDNA Synthesis Kit, RT was conducted, followed by PCR detection using SYBR Green I fluorescence method. AKT3 primer sequences: F: 5′-TGTGGATTTACCTTATCCCCTCA-3′, R: 5′-GTTTGGCTTTGGTCGTTCTGT-3′. 2^−ΔΔ*C*^_t_ was utilized to calculate the relative concentration of the samples to be tested. The same experiment was repeated three times for averaging.

### Detection via Western blotting

Total proteins were extracted by RIPA. On the basis of the molecular weight of target proteins, SDS/PAGE gel with appropriate concentration was selected. After electrophoresis, the proteins were transferred on to a PVDF membrane and dyed based on normal immune staining. Primary antibodies (diluted at 1:500) and secondary antibodies (diluted at 1:1000) were added for incubation at 4°C overnight and at 37°C for 2 h, respectively, followed by chemiluminescence, enhancement, fixing and photographing. Each experiment was repeated three times for averaging.

### Dual-luciferase reporter gene assay

It was predicted that the 3′-UTR sequence of AKT3 interacted with miR-16-5p, and pGL3 promoter vectors were injected with full-length AKT3 or a mutated sequence with the predicted target sites. Then the cells were inoculated on to a 24-well plate and co-transfected with pRL-SV40 (5 ng), a *Renilla* luciferase vector, to normalize the differences in transfection efficiency.

The article "MiR-16-5p inhibits breast cancer by reducing AKT3 to restrain NF-κB pathway" was retracted in 2022. Reasons: duplicated images; signs of a paper mill.

### Statistical analysis

Data were analyzed be means of SPSS20.0 and GraphPad statistical software, detected by the Student’s *t* test, and indicated by mean ± SD. *P*<0.05 indicated a statistically significant difference.

## Results

### Features and expression of miR-16-5p in breast cancer

Through the collection of clinical data of 72 patients with breast cancer in this center, it was discovered that compared with the high-expression miR-16-5p group, the low-expression miR-16-5p group had higher tumor classification (Table 1). Compared with that in paired adjacent noncancerous tissues, the expression of miR-16-5p in breast cancer tissues markedly declined (Figure 1A). Further, we found that miR-16-5p in breast cancer cells lines was prominently lower than that in MCF 10A cell line, in which the highest was in MCF-7 cell line and the lowest in BT-549 cell line (Figure 1B). Hence, MCF-7 and BT-549 cell lines were regarded as cell models in the following experiments. In the meantime, clinical data were assessed, which manifested that the survival rate of patients with highly expressed miR-16-5p was higher than that of patients with lowly expressed miR-16-5p (Figure 1C,D).

**Figure 1:** Features and expression of miR-16-5p in breast cancer (**A**) qRT-PCR detection results of the levels of miR-16-5p in breast cancer tissues (*n*=72) and paired adjacent noncancerous tissues (*n*=72) show that the level of miR-16-5p in the former is lower than in the latter. (**B**) The level of miR-16-5p in breast cancer cell lines is lower than in MCF 10A shown in qRT-PCR. (**C**) The level of miR-16-5p in the tumor tissues of patients with breast cancer displayed in qRT-PCR. (**D**) The survival rate of patients with highly expressed miR-16-5p is remarkably higher than in patients with lowly expressed miR-16-5p. The data are indicated as mean ± SD. *P≤0.05, Student’s *t* test.

**Table 1:** Patient clinicopathologic features

Clinicopathologic features	Number of cases	miR-16-5p expression		*P*-value
		Low (*n*=36)	High (*n*=36)	
Age				0.3061
<40	22	13	9	
≥40	50	23	27	
Tumor size				0.0177*
T1	40	15	25	
T2–T4	32	21	11	
N stages				0.0168*
N0	42	16	26	
N1–N3	30	20	10	
Metastasis				0.0244*
M0	64	29	35	
M1	8	7	1	

* denotes statistical significance.

### Cytobiological changes after treating cells with miR-16-5p mimics or inhibitors

We used miRNA mimics to up-regulate the expression of miR-16-5p in the cells and found that it was down-regulated by miRNA inhibitors (Figure 2A). EDU assay and CCK8 assay manifested that over-regulation of miR-16-5p can inhibit cell proliferation, and down-expression of miR-16-5p can promote it (Figure 2B,C). Through Transwell assay, we found that reducing miR-16-5p could facilitate cell migration, while overexpression of miR-16-5p could inhibit cell migration (Figure 2D). The cell cycle assay illustrated that overexpressing miR-16-5p could shorten the S phase, which could be prolonged by reducing miR-16-5p (Figure 2E). Through the cell apoptosis assay, we found that cutting miR-16-5p could reduce cell apoptosis, while overexpression of miR-16-5p could increase it (Figure 2F).

The article "MiR-16-5p inhibits breast cancer by reducing AKT3 to restrain NF-κB pathway" was retracted in 2022. Reasons: duplicated images; signs of a paper mill.

**Figure 2:** Cytobiological changes after cells were treated with miR-16-5p mimics or inhibitors (**A**) The level of miR-16-5p rises significantly after transfecting cells with miR-16-5p mimics, while down-regulation of miR-16-5p lowers the level of miR-16-5p. (**B**) CCK8 assay shows that reducing miR-16-5p promotes cell proliferation, but increasing miR-16-5p inhibits it. (**C**) EdU assay manifests that reducing miR-16-5p promotes cell proliferation, whereas elevating miR-16-5p suppresses it. (**D**) Transwell assay indicates that decreasing miR-16-5p stimulates cell migration, while overexpressed miR-16-5p inhibits it. (**E**) Cell cycle assays demonstrate that overexpressed miR-16-5p shortens the S phase, which can be prolonged by under-expressed miR-16-5p. (**F**) Cell apoptosis assays reveal that overexpression of miR-16-5p boosts cell apoptosis, while down-regulation of miR-16-5p has the opposite effect. The data are indicated as mean ± SD. *P≤0.05, Student’s *t* test.

### MiR-16-5p impedes breast cancer growth *in vivo*

After MCF-7 and BT-549 cell lines were subcutaneously inoculated, it was found that decreasing miR-16-5p could promote tumor growth *in vivo*. The tumor volume of cells with down-regulated miR-16-5p was bigger than NCs (Figure 3A), indicating that miR-16-5p impedes the proliferation of breast cancer cells *in vitro* and *in vivo*. MiR-16-5p inhibitor group had an evidently larger number of metastatic nodules on the lung surface than NC group (Figure 3B). Besides, it was verified by histological analysis that miR-16-5p reduced the incidence of lung metastasis in nude mice (Figure 3C).

**Figure 3:** MiR-16-5p promotes breast cancer growth *in vivo* (**A**) The tumor growth of mice in each group is detected after MCF-7 and BT-549 cell lines are subcutaneously inoculated (bar = 2 mm). (**B**) Metastatic nodes in lungs in different groups are counted after MCF-7 and BT-549 cell lines are injected through tail veins. (**C**) H&E staining images of lung tissues after MCF-7 and BT-549 cell lines are injected through tail veins (original magnification, ×200). The data are indicated as mean ± SD. *P≤0.05, Student’s *t* test.

The article "MiR-16-5p inhibits breast cancer by reducing AKT3 to restrain NF-κB pathway" was retracted in 2022. Reasons: duplicated images; signs of a paper mill.

### MiR-16-5p targets AKT3

According to qRT-PCR assay, the AKT3 expression in lesions was notably higher than that in paired adjacent noncancerous tissues (Figure 4A). We then used Western blotting experiments to verify this point (Figure 4B). It has been reported that the overexpression of AKT3 is involved in many cancers [21–23]. The luciferase reporter gene assays showed that miR-16-5p can be combined with AKT3 (Figure 4C,D). Furthermore, the AKT3 expression was revealed to be obviously elevated at the mRNA (Figure 4E) and protein levels (Figure 4F,G) after miR-16-5p inhibitors decreased the expression of miR-16-5p. Then we explored the expression of phosphorylated AKT3 (p-AKT3). Results showed that the changes of p-AKT3 in different groups are the same with total AKT-3 (Supplementary Figure S1A,B). It indicates that miR-16-5p targets AKT3, thus inhibiting the occurrence of breast cancer.

**Figure 4:** MiR-16-5p targets AKT3 (**A**) Comparison of the relative expression of AKT3 between breast cancer tissues and paired adjacent noncancerous tissues. AKT3 is markedly increased in breast cancer tissues. (**B**) Detection of the protein levels of AKT3 in breast cancer tissues and paired adjacent noncancerous tissues via Western blotting. (**C**) The putative miRNA binding sites in the AKT3 sequence. The putative miRNAs recognition sites is cloned downstream of the luciferase gene and named pGL3-AKT3-Wild. Bottom: mutations in the AKT3 sequence to create the mutant luciferase reporter constructs named pGL3-KT3-Mut. (**D**) The luciferase reporter in MCF-7 and BT-549 cell lines. Luciferase activity is determined using the Dual-luciferase assay and manifested as the normalization of the relative luciferase activity to *Renilla* activity. (**E**) miR-16-5p inhibitors are transfected into MCF-7 cells and the mRNA level of AKT3 is examined by qRT-PCR. (**F**) AKT3 protein levels in MCF-7 cells treated with miR-16-5p inhibitors or negative control are analyzed by Western blotting, with GAPDH as control. (**G**) AKT3 protein level in nude mice with tumor after MCF-7 cells treated with miR-16-5p inhibitors are implanted is analyzed via immunohistochemistry (IHC). The data are indicated as mean ± SD. *P≤0.05, Student’s *t* test.

### MiR-16-5p is reduced to block the NF-κB pathway

Reports have denoted that the abnormally activated NF-κB pathway participates in breast cancer [24]. After inhibitors were utilized to lower the miR-16-5p expression, the expression of P50 was prominently increased at the mRNA (Figure 5A) and protein levels (Figure 5B,C), and the expression of P65 exhibited the same trend at the mRNA (Figure 5D) and protein levels (Figure 5E,F). These results indicate that miR-16-5p is capable of decreasing the AKT3 expression and blocking the NF-κB pathway, so as to impede the onset of breast cancer.

The article "MiR-16-5p inhibits breast cancer by reducing AKT3 to restrain NF-κB pathway" was retracted in 2022. Reasons: duplicated images; signs of a paper mill.

**Figure 5:** Down-regulation of miR-16-5p promotes the pathway of NF-κB pathway (**A**) MiR-16-5p inhibitors are transfected into MCF-7 cells and the mRNA level of P50 is assessed by qRT-PCR. (**B**) P50 protein level after MCF-7 cells are treated with miR-16-5p inhibitors are examined via Western blotting, with GAPDH as control. (**C**) P50 protein level in nude mice with tumor after MCF-7 cells treated with miR-16-5p inhibitors are inoculated that are detected via IHC. (**D**) MiR-16-5p inhibitors are transfected into MCF-7 cells and the mRNA level of P65 is assessed via qRT-PCR. (**E**) P65 protein level after MCF-7 cells are treated with miR-16-5p inhibitors is analyzed via Western blotting, with GAPDH as control. (**F**) P65 protein level in nude mice with tumor after MCF-7 cells treated with miR-16-5p inhibitors are inoculated is examined via immunohistochemistry (IHC). The data are indicated as mean ± SD. *P≤0.05, Student’s *t* test.

## Discussion

Increasing show that miRNAs significantly contribute to the maintenance of normal cell growth and function, and changes in miRNAs expression has a close relationship to cancer [25–27]. It has been currently demonstrated that miRNAs suppress tumors [28]. For example, Okada et al. believed that miR-34 plays a tumor suppressive function by regulating p53 gene [29]. There are even reports that miRNAs can function directly as oncogenes [30]. Because miRNAs are involved in all kinds of important physiological processes, they have an important effect on homeostasis.

In the present study, in order to find the role of miRNAs in the occurrence of breast cancer, tissue samples were collected for experiments, which revealed that the miR-16-5p expression was remarkably under-expressed in breast cancer tissues compared with paired adjacent noncancerous tissues. Nevertheless, whether there are isoforms of miR-16-5p needs further exploration. We would perform Northern blot to verify it. Then, miR-16-5p mimics and inhibitors were used to transfect breast cancer cells, and the role of miRNA was examined via biological functional assays. Research has shown that miR-16-5p promotes the proliferation of tumor cells *in vivo* and *in vitro*, and tumor cells have strong migration ability. This ability is manifested as tumor metastasis in tumor development, whose degree indicates the malignancy of the tumor. In the present study, it was verified by cell migration assay that lowering the miR-16-5p expression can effectively increase the migration of tumors, indicating that under-expressed miR-16-5p in breast cancer patients can boost occurrence and migration of tumors. Among cell cycle, the SPF (S phase fraction) = S/(G_1_ + S + G_2_) reflects the proliferation activity of cells. The reduced miR-16-5p was found in the present study to remarkably increase the SPF. Apoptosis is a common process of cells, which regulates the growth and development of tissues and maintains the biological balance of the organism. Flow cytometry detection revealed that down-regulation of miR-16-5p could inhibit apoptosis of breast cancer cells, suggesting that low expression of miR-16-5p in breast cancer patients reduces apoptosis and triggers tumor. In a word, under-expressed miR-16-5p in breast cancer patients can effectively stimulate tumor cell migration and proliferation as well as DNA synthesis in the cycle, but impede cell apoptosis.

The article "MiR-16-5p inhibits breast cancer by reducing AKT3 to restrain NF-κB pathway" was retracted in 2022. Reasons: duplicated images; signs of a paper mill.

Subsequently, bioinformatics software such as REGRNA and TargetScan were jointly adopted for analysis to confirm that AKT3 is a potential target gene of miR-16-5p. AKT3 exhibits high expression in tumor cells, and its expression level is correlated with the pathological indexes including tumor occurrence, development, invasion and prognosis. Studies have confirmed that AKT3 may stimulate the occurrence of multiple tumors [31–33]. Therefore, we verified the combination of the miR-16-5p and AKT3 via luciferase reporter gene assay, and the results manifested that the expression of AKT3 was correspondingly elevated through down-regulation of miR-16-5p, proving that AKT3 is the potential target gene of miR-16-5p.

NF-κB/Rel protein contains NF-κB2 p52/p100, NF-κB1 P50/p105, c-rel, RelA/P65 and RelB that can act as polymerization transcription factor 2, modulate gene expression, and influence such biological processes as B cells and lymphoid organs formation, inflammation, innate and adaptive immunity and stress reaction [34]. The active NF-κB/Rel complex is further activated by post-translational modification and is transferred into the nucleus, alone or in conjunction with other transcription factors in the nucleus, including, Ets and Stat, AP-1 and mutually induces target gene expression [35,36]. In the alternative (or non-classical) NF-κB pathway, the NF-κB2 p100/RelB complex is inactivated in the cytoplasm. According to current studies, the activation of NF-κB pathway has a close association with the onset of breast cancer [37,38]. This study proved that miR-16-5p was involved in the mechanism of breast cancer by modulating the NF-κB pathway.

To sum up, it was found in the present study that miR-16-5p exhibited a low expression in breast cancer tissues, and the highly expressed miR-16-5p may impede the occurrence of breast cancer via modulating AKT3 and hindering the NF-κB pathway.

The article "MiR-16-5p inhibits breast cancer by reducing AKT3 to restrain NF-κB pathway" was retracted in 2022. Reasons: duplicated images; signs of a paper mill.

## Supporting information

**Supplementary Figure S1:** 

## Abbreviations

AKT3: AKT serine/threonine kinase 3
CCK8: Cell Counting Kit-8
EdU: 5′-Ethynyl-2′-deoxyuridine
FOXO1: forkhead box O1
HE: Haematoxylin and eosin
IHC: immunohistochemistry
NC: negative control
p-AKT3: phosphorylated AKT3
SPF: S phase fraction
